# Review on Hybrid Segmentation Methods for Identification of Brain Tumor in MRI

**DOI:** 10.1155/2022/1541980

**Published:** 2022-07-11

**Authors:** Khurram Ejaz, Mohd Shafry Mohd Rahim, Muhammad Arif, Diana Izdrui, Daniela Maria Craciun, Oana Geman

**Affiliations:** ^1^Department of Computer Science and Information Technology, The University of Lahore, Lahore, Pakistan; ^2^University of Technology Malaysia, Johor Bahru, Malaysia; ^3^Faculty of Physical Education and Sport, Stefan Cel Mare University of Suceava, Suceava, Romania

## Abstract

Modalities like MRI give information about organs and highlight diseases. Organ information is visualized in intensities. The segmentation method plays an important role in the identification of the region of interest (ROI). The ROI can be segmented from the image using clustering, features, and region extraction. Segmentation can be performed in steps; firstly, the region is extracted from the image. Secondly, feature extraction performed, and better features are selected. They can be shape, texture, or intensity. Thirdly, clustering segments the shape of tumor, tumor has specified shape, and shape is detected by feature. Clustering consists of FCM, K-means, FKM, and their hybrid. To support the segmentation, we conducted three studies (region extraction, feature, and clustering) which are discussed in the first line of this review paper. All these studies are targeting MRI as a modality. MRI visualization proved to be more accurate for the identification of diseases compared with other modalities. Information of the modality is compromised due to low pass image. In MRI Images, the tumor intensities are variable in tumor areas as well as in tumor boundaries.

## 1. Introduction

Medical imaging provides potential information and an easy visualization of diseases such as brain tumors to doctors and biomedical experts. The accurate identification of brain tumors requires a visualization of the disease area. Superior quality of visualization is possible on the MRI modality when the image processing technique or soft computing technique is used [1]. Tumor segmentation is possible with different soft clustering techniques and also with traditional image processing techniques. They help to identify accurate features for clinical analysis. Hence, segmentation techniques are helpful for the identification of the region of interest (ROI). The studies [2, 3] revealed that MRI faced numerous challenges for the identification of diseases.

Segmentation of medical imaging is not straightforward; it required sequence. Firstly, this was due to the MRI image being a low pass information image, and therefore more enhancements were required. Moreover, MRI dataset experiences data complexity issues. For cases of complex dataset, feature selection was required for the identification of relevant features for MRI images. Even though the images were enhanced, the ROI was still compromised due to the poorly managed intensities [4]. Moreover, although continuous tumor intensities were easy to detect, in certain situations, the segmentation process still requires special mechanisms for favorable results.

## 2. Related Work

In the comparative study, the literature of various previous studies was compared in terms of their efficient problem-solving capabilities. This comparative study is divided into three sections: (1) enhancement and region extraction, (2) feature reduction and selection, and (3) segmentation. Other literature studies have been considered for better segmentation results.

Here, image extraction is helpful as a pre-step in segmentation. Region extraction is also equally important. In a study, the pre-enhancement step is proposed where spackle noise is handled as compared to the Otsu algorithm. The study [3] preprocesses the image and handles the noisy images with localization. Noise of MRI image is tackled, region of interest is found out through feature extraction, and classification of cells is calculated [5]. In another study, different modalities were reviewed, and it was deduced that MRI segmentation is more challenging due to the low pass and high pass [6]. The confidence region is important to enhance the shape of a tumor with multiple parameters just like the classification of an image pixel to estimate the region of interest [7]. An improved Sobel edge detection algorithm, which draws close contour to extract the accurate region of a brain tumor, is proposed [3]. In this proposed algorithm, the bias correction field estimating the inhomogeneous intensities using two multiplicative components has a biased correction field and the input image. Reference [8] suggests that, for biomedical applications, software is used to check the active contour internal energy as well as external energy using the Marr, gradient vector flow, and vector field convolution methods [9]. In [10], a multilevel Otsu threshold enhances the image with determining 41 significant intensity points and assigns them threshold; then, using combination, they are enhanced by the algorithm.

In another study, an image enhancement was performed with denoising, watershed, and visual analysis of the image by connected components, and finally the image was evaluated [11]. A histogram was used as a formal analysis of the image, and the intensity of the brain tumor image was corrected by applying standard deviation.

In the given study, they mentioned the model about normalized the images, and obtained the information from the normalized image. The white portion in normalized image was enhanced and easily visible [12]. The MICCAI BraTS brain tumor dataset contained many aspects with a good set of data in comparison to other datasets. This processed brain tumor dataset then underwent a skull (cranium) stripping process of the image, where it was removed by the ITK tool kit [13]. Region scale fitting was enhanced where the edge stop function was improved. Hence, the region of interest denoises the noisy region [14]. In this study, the FCM was used to enhance the edges of the brain tumor image [15]. This method smoothly detected the inner contour versus the outer contour, while examining the start and end of the contour point. Hence, the background evolved smoothly from the foreground of the image [16]. There was a need for improvement of the edges of the brain tumor [17]. Furthermore, another study detected the edges of the region of interest (ROI) through the Bayesian contour, which also produced the measurement area and volume of ROI [11]. In another study, hyperintense lesion was dealt with through a combination of Gaussian mixture model, synthetic image, and support vector machine [18]. In [19], more focus has been made on the multi-contrast scan in which the variation of tumor stages is presented, 65 algorithms have been tested, and not a single algorithm has produced any good performance to classify the intensities properly. In addition, in another study, the accurate identification of a brain tumor was performed through the combination of growing region, segmentation, gray level cooccurrence matrix (GLCM) feature extraction, and classification through probabilistic neural network (PNN) [20, 21].

In [22], the enhanced Darwinian particle swarm optimization was compared with the PSO for the enhancement of the brain tumor image. The glioma tumor feature detection was classified using the Gaussian mixture model (GMM) in [23]. The initial learning rate improved the performance of self-organizing map (SOM) for the generation of a better dataset classification and results as suggested by [24]. Hence, the latest technologies have not improved the confidence region of brain tumor detection.

In the blow mentioned concepts, features like shape, texture, and intensity played an important role as an intermediate process between image enhancement and segmentation. Features were extracted from datasets, complex dataset values were classified, and hence classification features were able to be reduced. Therefore, the study needed certain feature selection criteria. The features were combined with other supervised and unsupervised algorithms. A better segmentation was achieved through the best texture-based feature by checking the entropy. With the SVM feature classification, the tumorous and nontumorous images were identified [25]. In [26], SOM was improved with its weights, and therefore its capabilities were improved for relevant feature selection. Furthermore, weighted SOM was improved at this level, and it did not require preprocessing. Furthermore, a higher classification accuracy feature was selected in [27]. Additionally, the study [28] contained accounts about the multiple kernels that selected the relevant features from the dataset. They were classified by SVM, and after the classification process, they assigned a label to each image with accuracy. In [24], there was an important step that was improved by using the Gaussian function that resulted in good performance. Another study [23] revealed that a Gaussian 43 mixture model showed the best feature accuracy on the heterogeneous tumor region as compared to the latest technology of PCA and wavelet. In [29], shape-based features were extracted with major axis, minor axis, area, circularity, and two-classifier decision tree algorithm, C4.5. The multilayer perceptron showcased the best classification accuracy. This kind of study was helpful in the analysis of image enhancement. At first, the image is segmented through the Berkeley wavelet algorithm. Next, the texture features were extracted and classified. The image was classified as tumorous and nontumorous accurately [30]. The major portion of [31] was about the analysis of an image labeled as tumorous and nontumorous. The first image was segmented through the execution of morphological operation, and the next image then underwent a texture feature extraction. Those extracted features were classified as tumorous and nontumorous.

In [31], the method was claimed to have improved the segmentation the Histogram of Oriented Gradients (HOGs) feature used to capture the variation of pixel values and these values are classified through the SVM. In [32], the segmentation was performed through the Spiking Pulse-Coupled Neural Network (SPCNN) with feature extraction through fast discrete curvelet transformation, reduction through PCA + LDA (linear discriminant analysis), and classification through probabilistic neural network. In [33], the features were extracted through two-dimensional discrete transformation wavelet and reduced through probabilistic principal component analysis, and the image was classified using AdaBoost algorithm. In [34], the classifier was improved where SWT was combined with PCA for dimension reduction, with four classifiers on SVM improved. In this referenced study, shape, texture, and intensity-based features were extracted, reduced, and classified. For feature reduction, principal component analysis was used. As the images hold high dimensionality, they will expand the computation time and the storage capacity. And they are classified as 2D extracted feature, whereas 3D extraction results in time consumption of 44 features [35]. In [36], multi-contrast images were analyzed through unsupervised algorithm, where efficient brain tumor structure was achieved [36]. In [37], numerous researchers cited here selected the optimal features with a combination of binary particle swarm optimization with mutation time variations. Additionally, in another study, the HOG feature-based classifier was suggested to detect brain tumor images [20]. Another study [38] revealed an updated self-organizing map, an improvement to SOM, which provided better feature classification as compared to the-state-of-the-art SOM. In [39], the nuclei-based neural network classified the tumor with the help of the proposed features. In [40], improved classification was proposed from the selected feature, and it was found to be helpful in the segmentation of brain tumor. Moreover, textural features were helpful for the detection of tumor types such as malignant or benign [41]. However, the review of the referenced studies showed that not a single study was able to select the best deterministic feature for segmentation.

Notably, segmentation is found to be a significant process for the exclusion of the tumor region in brain MRI. For segmentation, the detection of tumor-like feature is crucial, but the task is difficult especially when the intention is to detect a tumor automatically. The segmentation of medical images can be viewed by different methods. Surveys have been conducted to check both techniques of image processing under the umbrella of segmentation and different modalities of medical imaging [42]. Medical imaging is used for the analysis of image segmentation of the related 45 regions being analyzed, and it is based on different application techniques such as region-based, classification, or hybrid methods [43]. The segmentation can be also achieved through good statistical calculation, computational application on the dataset, and confusion matrix with its derivations [44]. It has been acknowledged that there is a conventional technique of segmentation which removes noise over boundaries of an MR image using filters [45]. Automatic segmentation becomes challenging if there are a variety of tumor tissues in the image [46]. Furthermore, in [47], an image was segmented through two phases. The first phase was to limit the image by using a histogram. The second phase involved the extraction of the tumor where an automatic seed was automatically adjusted. Hence, pixel-based segmentation was obtained [47]. In addition to these studies, image registration was a faster technique for segmentation as compared to active contour. In addition, with the cranium removal (skull stripped) image, the registration performance increases. The study [48] determined the complete enhancement of the tumor shape from a longitudinal analysis of the image. Moreover, this technique provided favorable results because of random regularization of image energy method applied. Therefore, extreme variation of intensities was easily managed [49]. In [50], a hyperintense MRI image FLAIR was used, and a small lesion was measured for clinical application. The small lesion was significant for the visualization of a small lesion of heterogonous shape of tumor. Based on [18], the heterogonous issue lies in the T2 weighted image, with the same intensity, a small lesion was also determined with the Gaussian mix model. This detection method identified the intensity outside the mean. In [51], three contributions were achieved; for one axial image, the brain's left and right parts were analyzed through unsupervised learning.

The second contribution was to enable the independent intensity normalization of an image, and the third was the segmentation of the brain tumor image through CNN. Multi-cascaded convolution neural network (MCCNN) with the combination of coarse fine-grain segmentation method produced a good segmentation, but these 46 segmentations were more enhanced with the connected conditional random field (CRF) [52]. In [53], the tumor was segmented using CNN and local as well as global features. With the reduction of the parameters, the issue of overfitting was also managed. The study was chosen to fine-tune the contour for registration. It enabled the descriptor extraction of an image block. Thus, adaptive matching was obtained. This process was a fully automatic process for the segmentation of brain tumors [54].

Another study explicated a two-phase process; in phase one, random forest algorithm generated a classified segmentation which was combined with the level set for delineation of the tumor boundaries [55]. This referenced method was good for the enhancement of the region of interest. It reduced the noise of signal-to-noise ratio. Firstly, the GLCM along with DWT was applied for denoising process. Then, a probabilistic neural network was used to identify the patch. After that, the segmentation analysis was made through classification [21]. The contrast resulting from the combination of criterion, fuzzy C-means and spatial technique produced an impactful segmentation. With this combination, the segmentation was addressed, and the outliner issue was also resolved [56]. In [1], the SOM performed initial clustering, which included the FKM and memberships at an average and soft computing techniques apart from artificial intelligence, which have been combined for new biomedical applications in present day. The soft computing techniques were then compared with their state-of-the-art techniques for performance measurement perspective.

Unsupervised learning plays an important role. According to [57], an unsupervised multi-objective algorithm was proposed. The target pixels were extracted in clusters. With the mentioned step, the region of interest (ROI) was segmented. According to [36], one unsupervised algorithm was applied for identification of contrast intensities. In comparison with the contrast, a deep learning neural network approach was proposed to segment region of interest (ROI); this practice of research was done for the purpose of automation, and the segmentation speed of the proposed algorithm was good for a number of brain tumor images. Manual practice was discouraged.

Different state-of-the-art literature exists; for example, [29] segments the tumor using deep learning neural network. U-Net is a deep learning model. This network was used for automation purpose. This automatic algorithm is compared with other state-of-the-art techniques. In another study [58], the 3D feature of images is taken as input, and then the input image is segmented through deep learning CNN. In another study, CNN 4.55 is combined with optimized parameters; CNN 4.55 is good for classification of the MRI feature; for more optimization, t-test is used for identification of the accurate classification parameter in disease image [58].

In [59], the K-means cluster is combined with morphological operation. The result of the combination of both techniques is segmentation of region of interest (inner information of tumor). In [60], a segmentation technique was suggested with combination of KFC and HCSD. KFCM segments the tumor pixel; this technique also gives the details of nontumorous pixels; however, HCSD segments the tumor pixel cluster. In another study, the tumorous pixels are extracted and then detected for accurate identification of accurate class of tumor cells in MRI images [61]. Twenty (20) matrices are evaluated to measure the accurate performance of the algorithm, fuzzy cluster values are compared with ground truth reality image, and then 20 parameters help to evaluate the results [62].

In line with the above study, three types of techniques, namely, hybrid-based technique, learning-based technique, and atlas-based technique, were used for the segmentation of tumor pixels, with the evaluation metrics being Dice and Jaccard [63]. In other research, the PSO and EDPSO are compared across 48 instances, and the results are verified for both classification and segmentation [22]. In another study, an unsupervised learning algorithm was proposed. The reason for the design of this algorithm was multiobjective.

In [64], both K-means and SOM are combined where SOM identifies the scattered pixel and K-means identifies hard clustering values of pixels. In [52], the multi-cascaded neural network offers portion segmentation. The multi-cascaded neural network with random forest was proposed, and this hybrid approach is compared with the random forest.

According to [53], the neural network is trained for segmentation using local and global feature. The results are improved with CNN parameter named as max pooling. In another study, contour was drawn around the boundaries of tumor for identification of tumor region [54]. In [56], a local based FCM algorithm (LCFCM_S) identifies the region with robust outlier. In another study, two phases are included for segmentation; in the first phase, voxel based classifier along with random forest is used, and in the second phase, active contours are identified using level set method (LSM) [55]. In addition, [65] reviewed the segmentation methods over MRI images.

In [66], the effective segmentation is performed through a series of steps. K-means cluster and FCM clusters are combined, the resultant cluster is further combined with morphological operation, and morphological operation is performed for thresholding of tumor pixels. In [42], different modalities like MRI and CT scan are discussed; these modalities can be further segmented and classified. In [1], traditional image processing is compared with soft computing. In [67], the segmentation of image is performed through K-means and analyzed through HOG feature along with SVM classifier for detection of brain image. An image was segmented by K-means segmentation with preprocessing of brain MRI.

In another study, the brain tumor image is segmented through combination of modified FCM (MFCM) and Bacteria Foraging Optimization (BFO) [68]. In [4], FKM is combined with SOM for identification of tumor boundaries, with the performance evaluation performed utilizing comparison parameters such as Dice overlap index (DOI), Jaccard index (JI), sensitivity, specificity, peak signal-to-noise ratio (PSNR), mean squared error (MSE), and computational time in addition to the memory needs for processing the magnetic resonance (MR) brain images. DOI and JI gave the voxel similarity, whereas the MSE and PSNR indicated the quality of image with numeric value. In this study, automatic detection of the tumor region in MR brain images was achieved and possessed a positive effect in assisting radio surgeons in identifying the precise topographical location of tumor region. In a study by Rahim et al. [69], local features were extracted for region detection, and eigenvectors were used for segmentation. Furthermore, in [70], a review was conducted on soft clustering, tradition image processing, and artificial neural network (ANN). In [71], it was revealed that automatic pathological analysis possessed greater value than manual image analysis, especially when the focus was on accuracy or time. In another study, a review was conducted to check the segmentation and evaluation methods for identification of disease [72]. In [63], for dedicated kind of method for MRI, segmentation of brain tumor (glioma) was suggested in a survey. In another study, a specific general classification-based segmentation was suggested with evaluation parameters like Dice and Jaccard.

In [73], segmentation is performed through deep learning on glioma images, and analysis of tumor is done through classification of glioma images as compared to normal cell images. In [74], a tumor is segmented through localization, then thresholding is performed, and at last statistical evaluation is performed. In [75], a study was conducted with a combination of SCM and modified SVM and modified FCM which provided a better segmentation of the brain tumor.

In another study, FLAIR sequence of MRI is segmented through the CNN technique. Another technique named as Simultaneous Truth Estimation (STAPLE) is used to generate the ground truth images. In [58], a cascade of 2.5D CNN was proposed for segmentation with classes of intensities of the brain tumor. In [76], very special deep learning technique, which assigns label to the global tumor images as compared to the detailed tumor image, was proposed. In [77], K-means is combined with CNN; in parallel for segmentation, the accuracy with unsupervised learning is more accurate as compared to supervised learning and CNN. In [78–84], segmentation methods are compared with deep learning. Hence, it is emphasized that not a single study among the referenced ones was capable of solving the issues of variation of intensities, extreme intensities, and features clustering.

In another study, efficient segmentation is performed with the combination of SOFM and FKM.

In studies like [85–91], segmentation and classification play an important role for identification of disease in medical imaging.

Figure 1 shows the design of the research process; this figure is a kind of pre-map of the review work. Furthermore, datasets of medical images are acquired. Then, those images are input to the preprocessing phase. In this phase, tumor region is extracted using the mentioned traditional image processing techniques. Furthermore, the higher-dimensional features of the big dataset images are reduced to small set. From small set, a set of specific features was selected through the mentioned techniques in Figure 1. The images of the big datasets are segmented through the preferred clustering techniques. All of the three phases are combined at the level of hybrid segmentation.

## 3. Dataset and Processing

Dataset and processing include the details of modalities like magnetic resonance imaging (MR). Modality information can be published or unpublished. It includes the details of MRI and MRI based dataset. The discussion can be seen in Section 3.1 and Section 3.2.

### 3.1. Magnetic Resonance Imaging (MRI)

Out of the different kinds of image modalities in existence, three modalities have been identified as being frequently used: the application of X-ray, computed tomography (CT), and magnetic resonance imaging (MRI). Notably, the MRI can be easily distinguished from the other two modalities. CT scan is more similar to MRI as both are able to view the internal structure of the physique. However, unlike MRI which utilizes a powerful magnet and radio waves to function, the CT scan employs a sophisticated X-ray system to capture a 360-degree image of the targeted internal body area and organs. The targeted human organ is exposed to the X-rays. During the process of CT scan, a person must be laid down on a sliding table, and the machine rotates for capturing cross-sectional images of the body. Meanwhile, X-rays utilize electromagnetic waves with a wavelength of approximately 0.01 to 10 nanometers. Pretibial *l* edema (PTE) indicates signs of abnormal level of fluid in the human body. All the three mentioned image modalities (X-ray, CT, and MRI) are medical imaging tests used in medical image processing. In medical imaging science, MRI is superior in many instances in comparison to X-rays and CT scan [92].

The main purpose of medical imaging is to process internal organ visualization. It is used to diagnose ailments. It is a must to possess prior knowledge regarding the chemistry of the human body before capturing images. A human body consists of matters termed as atoms. An atom consists of three elements: an electron, nucleus, and proton, where electrons revolve around the nuclei. Modalities give a powerfully aligned margin around the nuclei within the body.

The variable magnetic field inside the body that causes the atoms to resonate is called the nuclear magnetic resonance (NMR). The nuclei produce a strong magnetic field. The scanner detects the magnetic field and produces an image [42]. The MRI employs the same physical effect as the nuclear magnetic resonance (NMR).

The human body normally consists of water (H_2_0), composed of 2 hydrogen atoms (H_2_) and one oxygen atom. The hydrogen nuclei (protons) will align with the magnetic field of 0.2 to 3 tesla. The scanner produces a strong magnetic field that creates varying magnetic fields, and because protons are part of atoms, they will absorb varying energy from the variable field created by the scanner. They flip their spins when the field is turned off and gradually return to the normal spin which is called precession. The return of energy will produce a radio frequency that is measured by the receiver in a scanner, and this will create an image. The protons in the different parts of the body will return to their normal spin at different rates, and this enables the scanner to distinguish different tissues, assisted by the setting of the scanner which produces a contrast that enables this differentiation of the tissues. MRI is used for testing healthy and also abnormal cells and tissues with the use of microwaves that are spread over the internal organs of the human body to obtain an image of the targeted organ as shown in Figure 2.

In Figure 2, an MRI machine is presented with its components such as magnets that produce magnetic fields in the body, and the scanner will create the image. MRI provides magnetic field and X-rays such as radio frequency (RF) pulses; it is not recommended during radiation for the first diagnosis. For safety measures, the doctor goes through an MRI magnet. MRI uses an implanted magnet that heats up the field. Therefore, before the patient is examined, it is important to check and evaluate the implanted magnet properly and the patient's risk factors, for safety measures.

When a continuous magnetic ray is directed onto the patient, the ray penetrates through, and this sensation is felt by the patient. In addition, the flipping of a magnet used in MRI procedure produces a certain sound/beep noise; thus, for protection, it is necessary to insulate the room. The radiofrequency rays are transmitted by the scanner, and the body absorbs those radiations, thereby limiting the rays of the scanner. The future of the MRI with the advancement of science magnet flip has been modified, and now more magnets can be used. The enhancement of organ imaging with quantitative technique has enabled an image of the brain up to 1 mm be obtained. This permits doctors to perform analyses on brains.

Molecules tend to diffuse in a parallel manner along the fibers. A technique known as Digital Tensor Imaging (DTI) measures the parallel diffusion. Functional magnetic resonance imaging (fMRI) is a kind of MRI that checks the functional activity in the brain and measures the flow of blood toward other parts of the body. The fMRI basically measures the blood oxygen level depending on the contrast because the neurons of the body are active and contain more oxygen levels and vice versa. Most researchers employ the fMRI with DTI for examination and evaluation purposes. Nevertheless, for this current case study, the researchers ascertained that the MRI is adequate as the MRI quality of image is acknowledged to have undergone improvements. This current research study has identified the MRI as having sufficient accuracy to detect brain tumors, which is the focus of this study.

The brain tumor detection was realized through the modality of the MRI; an abnormal mass or cell collection in a particular part of the body is called a tumor. When this process is found in the brain, it is termed as a brain tumor. Furthermore, any tumor can be either benign (noncancerous) or malignant (cancerous). Both types have the potential to grow inside the brain, and their growth subsequently creates pressure within the brain, which is life threating. Brain tumors are classified into two main classes, primary and secondary. When tumors reside in the brain, they are termed as primary benign. When they spread to other parts such as the lungs and chest, they are termed as secondary tumors in which metastasis is formed, and this leads to the spread of the tumor. The risk factors of brain tumor are dependent upon age, race, family history, and race. The symptoms of brain tumors are vomiting, headache, confusion, and weakness.

Generally, doctors initiate their examination by checking the condition of the brain through the MRI. If a tumor is found, the doctor will then set out on further examination to determine whether the tumor is benign or malignant.

The MRI measures the size of the tumor in the brain after detailed imaging of the brain is executed. Before the imaging, a patient is given an injection into the vein which works as a tracer. The tracer helps to highlight the region of interest (ROI), which is ensued by detail MRI to detect a tumor.

T1 and T2 are important relaxation time factors as they can separate the tissues. The time constant for the *z*-axis plan is termed as the T1 parameter, whereas the time constant for the *xy*-axis plan is termed as the T2 parameter. T1 is greater than T2 element in the biological factor. T1 relaxation time difference produces a T1 weighted image, whereas the T2 relaxation time difference produces a T2 image. To determine the protons in every tissue, the sum of the protons in each tissue is taken per unit and is termed as proton density (PD) image.

During MRI, six items are employed with six components, and they are (1) coil, (2) shim coil, (3) radio frequency coil, (4) receiver coil, (5) gradient coil, and (6) computer. The CT scan and X-ay are both one-dimensional planes, whereas the MRI consists of three-dimensional planes. One of the dimensional planes consists of the axial plane, with the orientation of the image direction is from the head to feet. The next dimensional plane is the sagittal plane, with the orientation of the image plane from the back to the front of the human body. The third and final dimensional plane is the coronal *l* plane, with the orientation of the image plane from left arm to right arm. All of the images from the dimensional planes mentioned can be used for medical analysis of the internal body that enables doctors to perform clinical analysis. MRI does not perform ionization radiation. With short *T* relaxation time, fat signal typically appears bright in most significant clinical imaging sequences and can conceal the latent pathology such as edema, inflammation, or enhancing tumors. The visualization of the interior representation of a human body is akin to the internal tissues; it can be seen in Figure 2.

One of the disadvantages of the MRI images is the production of a noisy image. Occasionally, the image features are overlapped. In instances when a disease is discovered through the analysis of an image, the presence of overlapping features will pose problems to the clarity of the case. Furthermore, the MRI is considered as very expensive in comparison to modalities such as the X-ray. The aspect ratio of original image is 4 : 3. The most important benefit of MRI is its 3-dimensional image details.

The standard means of producing the information of the brain is using the brain imaging technique that presents the image of the brain in digital or MRI film format. There are many applied benefits of these images, for example, in clinical purposes such as diagnosis systems or forensic purposes such as human identification systems.

### 3.2. MRI Dataset

The MRI dataset can be found in both published and unpublished datasets. The published dataset is accessible online, whereas the unpublished ones need to be made available. Previously available published dataset is the Harvard brain tumor repository (such as https://www.med.harvard.edu/AANLIB/home.html). The main disadvantage of using this dataset images is the availability of skull (cranium) images. Presently available dataset is the MICCAI BraTS brain tumor dataset which consists of images of the brain with the exclusion of the skull (cranium) in the images [13]. Ground truth images are also available in the dataset. Scientists worldwide will enhance the dataset annually [19]. In Figures 3–6, four sequences of images are provided. They are termed as T1, FLAIR, T2, and T1CE. They indicate intensity-wise information in the dataset. They are also labeled based on their intensities. T1 provides the details of enhancing tumor core, while T2 and FLAIR provides the details of edema, and T1CE provides the details of enhancement as well as the complete shape of the tumor.

## 4. Approach

The segmentation and analysis of the brain tumor images with high accuracy using MRI are enabled through two methods, which are image processing and soft computing [94].

Image processing penetrates deep inside the tumor and is based on image information, whereas soft computing analyzes the image intelligently. With soft computing, the number of brain tumor image can provide the features of the image.  Figure 7 illustrates seven types of segmentations which are contour-based, region-based, multi-resolution-based, machine learning-based, and hybrid soft computing-based segmentations. Contour involves curve analysis of the shape. Region-based segmentation explores the information inside the edges. Statistical-based segmentation is used for investigation purposes and is divided into two groups; they are the clustering and the predictive modeling. Multi-resolution-based segmentation creates the objects through the employment of an iterative algorithm. Meanwhile, the machine learning techniques are used to divide the information of the image. However, different from the traditional techniques, soft computing employs the clustering techniques which provide information of the image; the techniques are combined in hybrid.

## 5. Image Enhancement

The term image enhancement refers to the improvement of the image appearance or to the improvement of the contrast and visibility of features of concern. In addition, image enhancement is the development of digital images to produce suitable results for analysis or demonstration; clustering gives particular information. These techniques perform the analyses of images. The enhancement of a medical image is important as it helps radiologists or surgeons to identify the abnormalities in human organs. The main medical image enhancement categories include the spatial domain methods and frequency domain methods.

Image enhancement provides brightness to an image by making changes in pixel values or by transformation of pixel values, and this has been accomplished with equations and formula. As Fourier transformation (FT) is also an example of image enhancement, the values of the pixel will be changed.

(1) $$\begin{array}{c} f⟶g, \end{array}$$

(2) $$\begin{array}{c} S=T\left(r\right). \end{array}$$

Equation (1) shows a one-to-one function, where *T* is the transformation of domain *f* to domain *g* with pixel, and the transformation pixels' intensity can be within the range [0–2k^−1^]. In (2), *T* is the transformation of *r* intensities. These intensities are formed with the mapping function. *S* is the variable in which the intensity values will be stored. Other transformations can enhance the image. Furthermore, *T* transformation has been used by logarithmic transformation, power transformation, and piece-wise linear image transformation and for intensity transformation of image [95].It can be seen in Figure 8 where one T1 image is input, and Figure 9 is the enhanced image.

## 6. Segmentation

In image processing, an image is an input, and after processing, the processed image is returned. The output is an image with attributes. The segmentation is carried out by subdividing an image into its parts or objects. This process of subdivision will be carried out till the problem is solved. Two properties of segmentation exist. These are continuous and discontinuous segmentation.

Segmentation can be seen by means of image processing and by soft computing. By using image processing, the intensity of detecting features is enabled by using line, edge, and point. The intensity of an image is also addressed through the soft computing methods. Some methods are represented in Table 1.

The segmentation methods are used for detecting features based on sharp local intensities and the type of feature that they can isolate such as edges, isolated lines, and isolated point edges which are found over the pixels where the intensity changes abruptly so as to reveal the connected edges of a pixel. An edge detector can be used to locate and identify an object. The line may be viewed as an edge segment in which the intensity of the background of either side is higher or lighter than the intensity of the line pixel. Points are line, and one point in width or height will be single pixel [95]. In the following paragraph, segmentation methods are discussed clearly by means of image processing and soft computing.

The study [97] indicated the cluster techniques K-means and fuzzy C-means (FCM) which were combined for tumor segmentation. The K-means functions rapidly, whereas FCM performs accurate segmentation of a brain tumor. Thus, the functions of these two techniques were combined to produce the K-means integrated with fuzzy C-means (KIFCM) approach, which was proposed for segmentation. Another study [74] of automatic segmentation of tumor from T2 is performed with statistical operation. This statistical-based segmentation enhanced the low intensities of an image. In addition, in a study [98] on a brain tumor detection method, the method involved the combination of steps such as preprocessing, segmentation through neural network, and image analysis that was performed though Gabor filter and Bayesian neural network classifier. In addition to the aforementioned studies, another study [2] revealed that the MRI was the widely preferred and used method of medical imaging. In this study, the statistical evaluation consists of the mean, median, mode, variance, and standard deviation. The mathematical *l* formulation was also discussed, where it facilitated the identification of the statistical features of an MRI image and aided the segmentation. In [99], the supervoxel (volume elements) was over-segmented. Congruent with this, the supervoxel of an image was compared to the supervoxel of the atlas (for multi-atlas segmentation of brain MR images). Accordingly, from the MRI supervoxel images, labels were transferred to the atlas. In another study [100], the automated localization of a brain tumor in the MRI that employed potential cluster was compared to the K-means clustering algorithm. The research suggested that future work could address the calculation of the appropriate number of N clusters to locate one or more tumors. This depends mainly on the relative total intensity of the tumor regions with respect to the total intensity of the image.

### 6.1. Segmentation Performance

The performance of an image processing algorithm is improved with segmentation. In the majority of studies, the image processing technique is combined with segmentation such as edge detection and is coupled with intensity thresholding. Image segmentation based on morphology is a good technique to be used for brain tumor identification. The segmentation techniques work with different types of image processing such as histogram equalization, filters, region of interest, classification, morphological operation, dominant gray level run length, feature selection, feature extraction, region growing, K-means clustering, expectation maximum, and fuzzy logic [41].

### 6.2. Threshold

Threshold is about mapping the intensity value of the corresponding pixel value. If TR is applied to pixels in the neighborhood yield and the (*x*, *y*) value of output, then *g* is equal to the neighbor with an origin at (*x*, *y*). Thus, segmentation directly focuses on the characteristics of an image such as region-based intensity and property.

#### 6.2.1. Threshold and Its Types

For the identification of intensity, consider a histogram T1. The histogram corresponds to the image in such a way that the background light and object pixels have intensity values that are grouped into two dominant modes. For global thresholding, *T* is constant over the image. For variable thresholding, T1 changes the image completely. It is also known that variable thresholding is also termed as local thresholding, where T1 at any point of the (*x*, *y*) can depend on the neighbor's mean of average. If T1 depends on the spatial coordinate of (*x*, *y*) in the variable thresholding, the term will be referred to as adaptive thresholding or dynamic thresholding. If the threshold problem involves certain histogram and the histogram has three threshold classes, one of the classes is for the background and two of the classes are for the objects; such classification is known as multi-thresholding classification.

#### 6.2.2. Region-Based Segmentation

The objective of segmentation is to partition an image into regions. The problem of finding boundaries of a region based on discontinuities is that the threshold is accomplished based on pixel distribution property, such as intensity via color. However, through advancements made in the field, segmentation of tumor region can be found directly [101].

A method known as region growing can assist in the identification of the seed based on the similarities of the neighboring pixels and on the predefined seeds. Seed selection is based on particular criteria. If there are no criteria available, then the study will compute each node and the same property of seed will be processed for region growing. The formation of clusters posits such a seed nearest to the centroid. There is a need for some descriptor based on certain color intensities or texture, or useful information. The descriptor will look for similar colors only, but not for their connectivity. Hence, the possibility for region growing is misleading.

Region growing will stop if no pixel satisfies the growth rate or due to the similarity of colors or texture. Therefore, considering the historical account of the pixel, it checks the likeness among the candidate pixels. Such a description is partially available [101].

#### 6.2.3. Histogram

In a histogram, an image in which the intensity levels are separately identified is generated. These intensity levels are derived from different ranges of pixel values. The complete ranges of intensities are available in the histogram. These intensities consist of a dynamic range which helps to increase the contrast of the gray scale level. Histogram equalization is the transformation of discrete distributive intensities into discrete distributive intensities. To normalize a histogram, each of its values is divided by the total number of pixels in an image. In histogram equalization, each value of the histogram is modified or the contrast of every value is calculated. It produces a linear trend to the cumulative distributive function (CDF) which is associated with the image. The processing of CDF relies on histogram equalization. Linear CDF results in a uniform histogram [102].

#### 6.2.4. Dominant Gray Level

This technique is mainly used for feature extraction. The dominant gray level run length matrix (DGLRLM) is based on the calculation or it is the computation of the gray level found in different channels or lengths. Different gray level run length or the different consequences of gray level run are applied in this study. Run length is used for segmentation; this technique is based on the gray level run, which is defined as a collinear that is connected to a set of pixels, all possessing the same gray level. The length of the run is the number of pixel points in every run or iteration [101].

#### 6.2.5. Range Filter

In the local subrange filter, statistical subrange of different intensities within the window was used. The range distance is the statistical measure of the sample variation. The edge is a discontinuity in mean intensity. If the variation in the local range is small, minor computation is needed. The local range distance is considered large if a region has large discontinuities at the intensity level. Hence, range filter detects the intensity values among the edges within the window. The output range may be max or min, where the range values are multiplied by a certain constant to affect a clear picture of edges. Local range filter needs less amount of time for execution because it has a small input as a range filter for segmentation through creating structure element for extraction of neighbor range value [47].

#### 6.2.6. Morphological Operation

The above-mentioned study was developed for binary images and later extended to the gray scale function and images. The fundamental morphological operations are erosion, dilation, opening, and closing. These operations are helpful to remove the cranium from the brain tumor image. They are very strong features of image processing. With these, the images' pixels can be added to or removed from the MRI image [101].

### 6.3. Feature Extraction

Feature extraction extracts the cluster that indicated the predicted tumor at the output. The extracted cluster is introduced to the threshold process. It may be the binary mask over the complete image. It makes the dark pixel darker and the white one whiter or brighter. In the threshold coding, each transformation coefficient is compared with threshold T2. If the value is less than that, it is compared with other thresholds and assigned zero. However, if it is more than threshold *T*, then it will be considered as effective.

The difference between feature selection and feature extraction is that for feature selection, the feature is of the subset of the original feature set. Meanwhile, in feature extraction, a new feature subset is built from the original one.

#### 6.3.1. Feature Selection

Feature selection is a process that selects a subset of features relevant to the application. With the help of feature selection, it enables the search for a subset of features in this study.

The criterion of selection is the extent of classification accuracy, based on the optimization subset of the feature chosen. This is performed for reduction of the data dimensions and computation time and an increase in the classification accuracy. The selection of a subset feature from the total number of features is based on the optimization criteria [43].

### 6.4. Feature Classification

A feature classification is considered as an important step in the medical imaging process for the identification of a brain tumor. There are various classifiers available. Based on the curtained phenomena, the extracted feature labels are evaluated. The K-means helps the accuracy of the feature classification. With the following studies, a critical discussion on feature classification will assist in the analysis for the best feature classification and their combination.

The ensuing discussion will be very helpful for the detection of brain tumor images. To detect brain tumors with MRI, it is important to achieve feature classification accuracy. Thus, if the accuracy has been achieved completely, then the accuracy from all of the three planes, namely, the *z*-axis termed as axial images of MRI, the *y*-axis image termed as the coronal plane, and the *x*-axis termed as the sagittal, is ensured.

In the prior discussion, classification and novel hybrid classifier were discussed for the detection of normal and abnormal brain incidences. In the majority of the studies, 100 per cent of classification accuracy is achieved after performing the experiments. In [103], a series of steps over image such as the wavelet transformation were performed. At different levels, features were then reduced by using principal component analysis (PCA) which is a dimensionality-reduction method for feature extraction. Finally, the backpropagation neural network (BP-NN) was employed, and it has been revealed that the accuracy over the axial *z*-axis images was more than 90 per cent. Henceforth, the modern classification and combinations of brain MRI images were invented. According to Zhang, [104], the proposed “weighted” type Fourier transformation (WFRFT) + principal component analysis (PCA) + generalize eigenvalue proximal SVM (GEPSVM), WFRFT + PCA_twin SVM (TSVM), indicated better results.

In addition, further advancements in the field brought forth the successful invention used for automatic abnormal brain detection that employed improved classifiers with the combination of quantum behaved particle swarm optimization (QPSO), kernel support vector machine (KSVM), and wavelet energy, obtaining the best results comparatively. Secondly, the wavelet energy feature was the best for abnormal brain detection through CAD (Computer Aided Diagnose) [105, 106]. After the application of a 5-fold cross validation technique, the KSVM PSO was applied over the trained data; optimal KSVM revealed the state of *t* normal or abnormal brain. Thus, this technique was applied to 90 images, with a 97.7 per cent accuracy, which is a higher accuracy in comparison to backpropagation neural network (BP-NN) (86.22%) and RBF-NN (91.33%) [107, 108]. In another study, for the automatic classification of brain MR images into normal or abnormal, the wavelet, SVM, and BBO were used. The results of this study showed comparatively better accuracy, 97.78 per cent, than that of other studies using the biogeography-based optimization.

KSVM (BBO-KSVM) technique [105] is a combination of biogeography-based optimization and particle swarm optimization, and it is used to train the FNN. In [107], the stationary wavelet transformation (SWT) produced better results. The classification results were 98.5 per cent with a combination of adaptive comparative particle swarm optimization (ADCPSO) and fuzzy neural network (FNN) derived from over 160 images from the Harvard site, and neural network has been applied [107]. Scalable Chaotic Artificial Bee Colony algorithm classifies normal and abnormal brains of T1 weight images with an accuracy of 100 per cent [109]. In [110], automatic detection of tumorous and nontumorous images was performed with 99 per cent accuracy through the combination of DWT, PCA, and LS classifier. An automated and intelligent medical decision support system is in use for brain MRI scan classification. Hence, the optimal classifier combination demonstrated a higher classification accuracy of MRI brain tumor images for identification. In Table 2, a combination of feature extraction, reduction, selection, and classification is given. From the abovementioned details, their classification accuracy can be observed.

#### 6.4.1. Overlap Accuracy (OA)

Overlap accuracy is determined by the statistical measure where the closeness of an image or object is measured. The overlap accuracy calculates the extent of the overlap of the white portion and how much overlap of the white portion occurs among two images of black and white. One image is a ground truth reality image, and another image is a segmented image. It is determined that images have complete overlap when the segmented image perfectly matches the ground truth reality image. With black and white input images where foreground is white and background is black, the conditions are as follows: If the segmented foreground white pixels overlap with the ground truth of the foreground, the image will then be considered as true positive, and the pixels will be labeled as foreground and indicate the tumor portion. In another case, the background portion will show up as black pixels of the tumor image when they overlap with the background black pixels of the ground truth image, where the image will then be considered as true negative. When the foreground pixels in the segmented image overlap with the background of ground truth, the image will then be considered as false positive. In another case, when the segmented image background overlaps with the foreground of ground truth reality image, the image will be considered as false negative.

(3) $$\begin{array}{c} A=\text{segmented image}, \end{array}$$

(4) $$\begin{array}{c} B=\text{ground truth reality image,} \end{array}$$

(5) $$\begin{array}{c} \text{total image area}=A*B, \end{array}$$

(6) $$\begin{array}{c} OA=\left(\frac{\text{total image area}}{A}\right)*100. \end{array}$$

Equation (3) is the segmented or the test image, and this segmented image is stored in A. Equation (4) shows the ground truth reality image, and it is stored in variable B. The total image area is the product, and this is shown in (5) and is formed with the combination of (3) and (4). Finally, (6) returns the percentage of the overlap of the white foreground segmented pixel with the white foreground ground truth pixel and is formed with the combination of (3) and (4).

## 7. Discussion

From the content of the article, it was found that region extraction, feature selection, and hybrid segmentation were the most applied methods. They played important roles in medical image processing (MIP). Similarly, better techniques have been proposed in the field of MIP. However, MIP was still lacking in areas pertaining to region extraction, confidence element extraction, and segmentation; therefore, time was needed to invent new methods or extend existing ones. Notably, dataset is an important element in the field of MIP. Datasets like Harvard brain tumor repository and BraTS brain tumor challenge are helpful for experimentation. A huge amount of experimentation has been performed, but issues persist and were visualized when the sequence of image (FLAIR, T1, T2, T1CE) was analyzed. In BraTS brain tumor dataset, the tumor core region was enhanced by the T1 sequence; thus, it is important to analyze this region. It can be seen in article [20] that the edema region, complete tumor region, and enhancing tumor region show the tumor areas with different labels. Due to the intensities, a labeled image seems to be challenging.

The scope of the mentioned issues is crucial, as the issues are opening new horizon which needs inventions and improvements. Firstly, the MRI image region extraction was executed through confidence interval, but it was inadequate for the identification of complete tumor pixels. These pixels are required in enhancing tumor core. If tumor pixels can be identified, the probability of tumor region identification increases. Therefore, in [111], the confidence region was needed for the accurate identification of enhancing tumor. Secondly, in another suggested study, SOM selection assigned weight to the features, but improvement was required to select the best single feature. These features must be highly accredited feature on the dataset. Due to the high cost of processing, the feature selection algorithm needed improvement. Accurate features are needed to assist in the segmentation of tumors [26].

In some other studies, hybrid segmentation algorithm was used. Segmentation was achieved, but extreme variations or extending intensities of intensity were an open question. Extreme intensities of tumor were mixed with other normal brain intensities [52]. Therefore, there were issues in the hybrid segmentation methods when the algorithm performed segmentation. A hybrid unsupervised learning algorithm was required for managing the extreme variation of intensities [68].

## 8. Conclusion

MRI modality is compared with other modalities like CT scan, X-rays, and PET scan. Different state-of-the-art studies over brain tumor detection are available, like, feature selection and segmentation technique. Where the region extraction techniques identifies region of brain tumor and features are extracted and selected from the image dataset. Segmentation gives region of interest after series of steps. Concepts are more specific on MRI like MR imaging, MRI dataset, MRI enhancement, segmentation, feature extraction, comparative studies, and discussion on the basis of critical analysis. We can see after comparative analysis of techniques that the article highlights issues of variation of intensity, which needs to be extracted from a certain region of brain; secondly, feature selection is important aspect from big datasets, and the specific feature selection from state of the SOFM is another challenge. Finally, segmentation is required for extreme variation of intensities on the tumor boundaries.

## Figures and Tables

**Figure 1:** Process of medical image segmentation.

**Figure 2:** Architecture of MRI machine (source: [93]).

**Figure 3:** Image of T1 (BraTS17_13_2_1).

**Figure 4:** Image of FLAIR (BraTS17_13_2_1).

**Figure 5:** Image of T2 (BraTS17_13_2_1).

**Figure 6:** Image of T1CE (BraTS17_13_2_1).

**Figure 7:** Soft computing and image segmentation approaches.

**Figure 8:** Input T1 sequence image.

**Figure 9:** Image enhancement of Figure 8.

**Table 1:** Segmentation techniques.

Sr. no.	References	Techniques
1	[96]	Histogram, fuzzy c-means, and K-means
2	[42]	Thresholding, region growing, clustering, classifiers, Bayesian approach, deformable methods, atlas guided approach, edge-based methods, and compression-based method
3	[43]	Thresholding, histogram, region of interest (ROI), clustering techniques, classification techniques, expectation maximization, and graph cut
4	[45]	Image texturing and range filters
5	[46]	Dominant gray level run length

**Table 2:** Combination of classification technique and classification accuracy.

Sr. no.	Referenced studies	Techniques
1	[103]	DWT, SWT
2	[105]	Artificial B colony algorithm DWT
		PCA K-fold stratified cross validation FNN classifier
		SCAB
3	[107]	Fourier transformation, DWT, BNN
4	[110]	DWT, PCA, SVM
		Kernel-SVM (KSVM)
		K-fold technique

## Data Availability

No data were used to support this study.
